# Modeling and Optimization of Water Distribution in Mineral Processing considering Water Cost and Recycled Water

**DOI:** 10.1155/2022/2314788

**Published:** 2022-02-01

**Authors:** He Wang, Qiuyu Cui, Hualong Du

**Affiliations:** School of Mechanical Engineering and Automation, University of Science and Technology Liaoning, Anshan 114051, China

## Abstract

Reducing mineral processing water costs and freshwater consumption is a challenging task in the mineral processing water distribution (MPWD). The work presented in this paper focuses on two aspects of the MPWD optimization model and the MPWD optimization method. To achieve MPWD optimization effectively, a nonlinear constrained multiobjective model is built. The problem is formulated with two objectives of minimizing the mineral processing water costs and maximizing the amount of recycled water. In this paper, an optimization method named enhancing the multiobjective artificial bee colony (EMOABC) algorithm is proposed to solve this model. The EMOABC algorithm uses four strategies to obtain the Pareto-optimal solutions and to achieve the MPWD optimal solutions. With the three benchmark functions, the EMOABC algorithm outperforms the other two widely used algorithms in solving complex multiobjective optimization problems. The EMOABC algorithm is then applied to two cases. Results have shown that the proposed algorithm has the ability to solve the MPWD optimization model. The developed model and the proposed algorithm provide decision support for the actual MPWD problem.

## 1. Introduction

Mineral processing is the process of obtaining the raw materials for smelting and consumes large amounts of water. For water distribution, the decision-makers in mineral processing plants need to make decisions concerning different objectives, such as water costs and freshwater minimization, to maximize the comprehensive benefits of mineral processing plants. The solution to the multiobjective optimization problem often results from both an optimization model and an optimization algorithm. Thus, this paper focuses on solving mineral processing water distribution (MPWD) optimization problems from these two perspectives.

Over the years, many works have examined the water distribution optimization problem and presented many mathematical models and conventional methods such as linear programming [1, 2], nonlinear programming [3], and integer linear programming [4], which have been applied to solve the problem. However, these methods suffer from severe limitations in handling discreteness, nonlinearity, complex constraints, and local convergence [5]. To overcome the limitations of classical optimization methods, the heuristic methods have been proposed to solve water distribution optimization, such as simulated annealing (SA) algorithms [6, 7], genetic algorithms (GA) [5, 8, 9], differential evolution (DE) algorithms [10–12], particle swarm optimization (PSO) [13–15], ant colony optimization (ACO) [16–18], strength Pareto evolutionary algorithm (SPEA) [19], and shuffled frog leaping algorithm (SFLA) [20, 21]. Despite the success of these heuristic methods in certain aspects, they have not been applied to solve MPWD problems. Currently, MPWD problems are mainly based on manual scheduling. Therefore, building MPWD model and applying heuristic methods to solve the model represent an important issue of our current concern.

Heuristic methods have been widely used in various fields [22–25]. The artificial bee colony (ABC) algorithm is a relatively new heuristic method that has been proven to be an excellent competitor in multiobjective problems [26]. Several multiobjective ABC algorithms (MOABCs) have been proposed for multiobjective problems [27–29]. However, compared to the huge in-depth studies of other heuristic methods, such as nondominated sorting genetic algorithm II (NSGA-II) [30] and multiobjective particle swarm optimization (MOPSO) [31], on multiobjective problems, improving the performance of MOABCs is still a challenge.

MPWD is a complex process in which interrelated factors are multiple. In addition to meeting the total amount of mineral processing water, many factors, such as the flow of the water source, the pressure of the water source, and maximizing the use of recycled water, need to be considered. The traditional linear model is difficult to describe the relationship between these complex factors for MPWD with the above characteristics and cannot treat multiple constraints appropriately.

The purpose of this paper is to build a nonlinear and multiobjective model for MPWD and to develop an MOABC algorithm for solving the MPWD optimization problem. The MPWD optimization model has two objectives: one objective is to minimize mineral processing water costs, and the other objective is to maximize the amount of recycled water. The proposed MOABC algorithm called enhancing multiobjective artificial bee colony (EMOABC) algorithm integrated multiple strategies to improve its performance. Therefore, some of the contributions of this paper are as follows:

1. The developed model for MPWD is the nonlinear model that has two objective functions
2. The proposed EMOABC algorithm can improve the population diversity and obtain better global convergence

The rest of the paper is organized as follows: In Section 2, the MPWD optimization model is built.  Section 3 first gives a review of the basic ABC algorithm and then proposes the EMOABC and presents the results of the EMOABC algorithm compared with other algorithms on three widely used benchmark functions. In Section 4, the implementation of the EMOABC on the MPWD optimization problem is presented.  Section 5 outlines the conclusions.

## 2. MPWD Model

According to categories of water source, the mineral processing water can be divided into fresh water，tailings water, clean water, and in-plant water, and they are from rivers and lakes, tailings reservoirs, wastewater treatment plants, and in-plant recycled systems, respectively (Figure 1). The cost of using the tailings water, the clean water, and in-plant water is relatively high for proper treatment and long-distance transmission before entering into the mineral processing plant. Although the cost of using fresh water is very low due to no treatment required, it is important to minimize the use of fresh water for environmental reasons. Mineral processing water becomes wastewater after mineral processing. The MPWD problem in this paper is to optimize two competing objective functions simultaneously, minimizing the mineral processing costs and maximizing the amount of recycled water including tailings water, clean water, and in-plant water, while satisfying several equality and inequality constraints. Generally, the problem is formulated as follows.

### 2.1. Decision Variable

The vector of the mineral processing water is expressed as **Q**, including the freshwater as **Q**_**1**_, tailings water as **Q**_**2**_, clean water as **Q**_**3**_, and in-plant water as **Q**_**4**_. The mineral processing water except freshwater is called the recycled water. The vector of the recycled water is expressed as **Q**′={**Q**′*| ***Q**_**2**_ ∪ **Q**_**3**_ ∪ **Q**_**4**_}. *q*_*i*_ is a flow of the *i*th water source; *a*, *b*, *c*, and *n* are positive integers, and *n* is the number of water sources. Decision variables are defined as follows:

(1) $$\begin{array}{c} Q=\left(q_{1},q_{2},\ldots ,q_{n}\right),\\ Q_{1}=\left(q_{1},q_{2},\ldots ,q_{a}\right),\\ Q_{2}=\left(q_{a+1},q_{a+2},\ldots ,q_{b}\right),\\ Q_{3}=\left(q_{b+1},q_{b+2},\ldots ,q_{c}\right),\\ Q_{4}=\left(q_{c+1},q_{c+2},\ldots ,q_{n}\right). \end{array}$$

### 2.2. Objective Function

Let *c*_i_ be the cost coefficient of the *i*th water source; its meaning is the total power consumption required to lift one meter per unit volume of water. Then the mineral processing water costs in a certain hour are expressed as

(2) $$\begin{array}{c} C\left(Q\right)=\sum_{i=1}^{n}c_{i}q_{i}\left(100p_{i}+h_{i}\right), \end{array}$$

where *h*_*i*_ is the elevation difference of the *i*th water source; the integer 100 is used for unit conversion. *p*_*i*_ is the pressure of the *i*th water source. Equation (2) also can be transformed into

(3) $$\begin{array}{c} C\left(Q\right)=\sum_{i=1}^{n}c_{i}q_{i}\left[100f\left(q_{\text{sum}},q_{i},q_{i}q_{j}\right)+h_{i}\right], \end{array}$$

where *f*(*q*_sum_, *q*_*i*_, *q*_*i*_*q*_*j*_) is the macro model of the water supply network. This *q*_sum_ is the total flow of mineral processing water required in the mineral processing plant.

The yields of freshwater are low, but its prices are high. So it is important for cost reduction that the recycled water is used in mineral processing. While the total water consumption of mineral processing is met, the recycled water should be used in mineral processing as much as possible. The amount of the recycled water used in mineral processing can be expressed as

(4) $$\begin{array}{c} M\left(Q^{\prime }\right)=M\left(q_{a+1},q_{a+2},\cdots ,q_{n}\right)=\overset{b}{\underset{i=a+1}{\sum }}\alpha_{i}q_{i}+\overset{c}{\underset{i=b+1}{\sum }}\beta_{i}q_{i}+\overset{n}{\underset{i=c+1}{\sum }}\chi_{i}q_{i}, \end{array}$$

where *α* is the penalty factor of tailings water; *β* is the penalty factor of clean water; and *χ* is the penalty factor of in-plant water.

### 2.3. Constraint Condition

The sum of the flow from the water source should be equal to the total flow of mineral processing water required in mineral processing:

(5) $$\begin{array}{c} \sum_{i=1}^{n}q_{i}=q_{\text{sum}}. \end{array}$$

Each water source should be between the maximum and minimum water supply capacity:

(6) $$\begin{array}{c} \begin{array}{cc} q_{i}^{\min}\leq q_{i}\leq q_{i}^{\max} & i=1,2,\cdots ,n \end{array}, \end{array}$$

where *q*_*i*_^max^ and *q*_*i*_^min^ are upper and lower limits for the flow of the *i*th water source.

To ensure efficient transmission, the output pressure of each water source should be restricted as follows:

(7) $$\begin{array}{c} \begin{array}{cc} p_{i}^{\min}\leq p_{i}\leq p_{i}^{\max} & i=1,2,\cdots ,n \end{array}, \end{array}$$

where *p*_*i*_^max^ and *p*_*i*_^min^ are upper and lower limits for the pressure of the *i*th water source. Equation (7) also can be transformed into

(8) $$\begin{array}{c} \begin{array}{cc} p_{i}^{\min}\leq f\left(q_{\text{sum}},q_{i},q_{i}q_{j}\right)\leq p_{i}^{\max} & i=1,2,\cdots ,n \end{array}. \end{array}$$

To ensure the pressure requirements of the mineral processing plant, there should be a lower limit for the pressure at the control point.

(9) $$\begin{array}{c} \begin{array}{cc} {\text{cp}}_{i}\geq {\text{cp}}_{i}^{\min} & i=1,2,\cdots ,n \end{array}, \end{array}$$

where cp_*i*_ is the pressure at the control point of the *i*th water source; cp_*i*_^min^ is lower limit for the pressure at the control point of the *i*th water source. Equation (9) also can be transformed into

(10) $$\begin{array}{c} \begin{array}{cc} f^{\prime }\left(q_{\text{sum}},q_{i}\right)\geq {\text{cp}}_{i}^{\min}, & i=1,2,\ldots ,n \end{array}, \end{array}$$

where *f*′(*q*_sum_, *q*_*i*_) is the macro model of the pressure control point.

### 2.4. Final Model

In summary, the water optimization model for the mineral processing plant is a two-objective optimization model and its final model is expressed as follows:

(11) $$\begin{array}{c} \min\left\{C\left(Q\right)\right\},\max\left\{M\left(Q^{\prime }\right)\right\},\\ \text{s}.\text{t}.\left\{\begin{array}{c} \sum_{i=1}^{n}q_{1}=q_{\text{sum}},\\ q_{i}^{\min}\leq f_{i}\leq q_{i}^{\max},\;i=1,2,\ldots ,n,\\ p_{i}^{\min}\leq f\left(q_{\text{sum}},q_{i},q_{i}q_{j}\right)\leq p_{i}^{\max},\;i=1,2,\ldots ,n,\\ f^{\prime }\left(q_{\text{sum}},q_{i}\right)\leq {\text{cp}}_{i}^{\min},\;i=1,2,\ldots ,n. \end{array}\right. \end{array}$$

## 3. Enhancing Multiobjective Artificial Bee Colony Algorithm

With the above model and constraints, the appropriate optimization algorithm is applied to optimize the MPWD problem. In this study, an EMOABC algorithm was proposed to solve the developed MPWD model.

### 3.1. Basic ABC Algorithm

ABC algorithm is a swarm intelligence optimization method proposed by Karaboga to simulate the process of bees searching for nectar [32]. In the framework of the artificial bee colony algorithm, the location of the food source represents the possible candidate solutions of the problem to be optimized, the number of nectars in the food source represents the fitness (objective function value) corresponding to the candidate solutions, and the size of the bee colony is equal to the number of solutions. The basic structure of the ABC algorithm can be divided into the four following stages.

The first is initial stage, where ABC algorithm randomly generates a matrix **X** = [*x*_ij_]_*N*×*D*_, *N* is the population size and represents the number of candidate solutions, and *D* is the number of solution parameters, *i* ∈ (1, 2,…, *N*), *j* ∈ (1, 2,…, *D*). *D*-dimensional vector **X**_**i**_ = [*x*_*i*1_, *x*_*i*2_,…, x_*iD*_] is one of the candidate solutions. *x*_ij_ are randomly generated by

(12) $$\begin{array}{c} x_{\text{ij}}=x_{j}^{\min}+{\text{rand}}_{j}\left(x_{j}^{\max}-x_{j}^{\min}\right), \end{array}$$

where *x*_*j*_^max^ and *x*_*j*_^min^ are the upper and lower bound constraints of the *j*th variable of **X**_**i**_, respectively, and rand _j_ is a uniformly distributed random number within the range [0, 1].

The second is employed bee stage, where an employed bee is to modify and generate a new candidate solution based on the currently collected information, as well as to calculate its fitness. If the fitness of the new candidate solution is higher than the fitness of the original candidate solution, the new candidate solution replaces the original candidate solution; otherwise, the original candidate solution is retained. After all employed bees complete the search task, they share the information on the location of the food source (candidate solution) and the amount of nectar (fitness) they found with onlooker bees. The new candidate solution is generated by

(13) $$\begin{array}{c} v_{ij}=x_{ij}+\varphi_{ij}\left(x_{ij}-x_{kj}\right), \end{array}$$

where *k* and *j* are randomly chosen indexes, *k* ≠ *i*. *φ*_*ij*_ is a random number in the range [−1, 1]. The fitness of a solution can be defined as

(14) $$\begin{array}{c} \text{fit}\left(X_{i}\right)=\left\{\begin{array}{c} \begin{array}{cc} \frac{1}{1+f\left(X_{i}\right)}, & \text{if }f\left(X_{i}\right)>0, \end{array}\\ \begin{array}{cc} 1+\left|f\left(X_{i}\right)\right|, & \text{if }f\left(X_{i}\right)\leq 0. \end{array} \end{array}\right. \end{array}$$

The third is onlooker bee stage, where onlooker bees assess the fitness of candidate solutions passed from the employed bee and then select food sources based on the probability corresponding to the amount of nectar. In this case, the onlooker bee updates the candidate solution based on the original candidate solution and calculates its fitness; if the fitness of the new candidate solution is higher than the original candidate solution, the new candidate solution replaces the original candidate solution; otherwise, the original candidate solution is retained. The probability of a food source chosen by an onlooker bee can be calculated by

(15) $$\begin{array}{c} p_{i}=\frac{\text{fit}\left(X_{i}\right)}{\sum_{i=1}^{N}\text{fit}\left(X_{i}\right)}. \end{array}$$

The fourth is scout bee stage; if the nectar of the discovered food source is too inferior to find better solutions several times in a row (“*limit*” is denoted as the maximum number of times), it will be replaced by a new food source that a scout bee randomly found, and then the new food source is generated by (12).

### 3.2. Proposed Method

This section presents a detailed description of the proposed EMOABC algorithm. It can be observed from the literature that this approach to mineral processing water has not yet been extensively explored.

Inspired by the idea of NSGA-II algorithm [30] and DNSPSO algorithm [33], in this paper, the EMOABC is integrated with a series of multiobjective optimization strategies. It includes four important multiobjective strategies: noninferior ranking strategy, Pareto-optimal strategy, crowding distance strategy, and search strategy to evaluate the food source location multiobjectively and select the nondominated solution, so they are presented as follows:

(1) Noninferior ranking strategy: all individuals in the population that are not dominated by other solutions (noninferior solutions) are defined as rank 1; that is, the virtual fitness of the individual is 1; then these individuals are removed from the population, and new noninferior solutions are identified from the remaining individuals, which are defined as rank 2; that is, the virtual fitness of the individual is 2; the above process is repeated until all individuals in the population have been assigned the corresponding rank. By storing the current solution and all the individuals in the population in a hierarchical manner, the high-performance individuals can have a higher probability of survival and the population rank can be improved rapidly.
(2) Pareto-optimal strategy: the Pareto set is multiple viable solutions, which can provide multiple viable solutions in the supply of water to the mineral processing plant and can also reduce supply efficiency. Manual Pareto selection suffers from a variety of subjective uncertainties, which can make the selected solution less than optimal.
Define a function *η*_*i*_, representing the proportion of the *i*th objective function value of a solution in the Pareto set that is located along the direction of that objective function in front of the Pareto. The function *η*_*i*_ is expressed as
  (16) $$\begin{array}{c} \eta_{i}=\left\{\begin{array}{c} \begin{array}{cc} 1, & V_{i}\leq V_{i}^{\min} \end{array}\\ \begin{array}{cc} \frac{V_{i}^{\max}-V_{i}}{V_{i}^{\max}-V_{i}^{\min}}, & V_{i}^{\min}\leq V_{i}\leq V_{i}^{\max} \end{array}\\ \begin{array}{cc} 0, & V_{i}\geq V_{i}^{\max} \end{array} \end{array}\right., \end{array}$$
where *V*_*i*_^max^ and *V*_*i*_^min^ are the maximum and minimum values of the *i*th objective function in the Pareto set, respectively; *V*_*i*_ is the function value of the *i*th objective function. For each noninferior solution *k*, the normalized membership function *ƞk* is calculated by the following equation:
  (17) $$\begin{array}{c} \eta^{k}=\frac{\sum_{i=1}^{N_{ob}}\eta_{i}^{k}}{\sum_{j=1}^{M}\sum_{i=1}^{N_{ob}}\eta_{i}^{j}}, \end{array}$$
where *M* is the number of noninferior solutions in the Pareto set, and *N*_ob_ is the number of objective functions. The larger the value of *ƞk*, the better the performance of *k* in coordinating multiple objective functions. Sorting the Pareto set by the *ƞk* value gives a priority sequence of noninferior solutions.
(3) Crowding distance strategy: the crowding distance is used to estimate how dense a solution is with other solutions around it. For each objective function, the set of noninferior solutions is sorted by the objective function value; then, for each solution *x*, the sum of the two sides of the rectangle formed by the solutions *x* + 1 and *x* − 1 is calculated; the final result is the crowding distance *x*_dist_ of the solution *x*. The crowding distance of the boundary solution is infinite. When two solutions have the same rank (i.e., the same virtual fitness), the superiority of the two solutions can be compared by the crowding distance. It can be seen that *x* individual is superior to *y* individual when and only when *x*_rank_ < *y*_rank_ or *x*_rank_ = *y*_rank_ and *x*_dist_ > *y*_dist_.
(4) Search strategy: as one of the most representative variants, DNSPSO algorithm is characterized by introducing a global NS operator [33]. Therefore, the search strategy in this paper also adds that operator, and it can be expressed as follows:
  (18) $$\begin{array}{c} v_{ij}=r_{1}x_{ij}+r_{2}x_{\text{best}}+r_{3}\left(x_{aj}-x_{bj}\right), \end{array}$$
where *r*_1_, *r*_2_, and *r*_3_ are three mutually exclusive numbers which are randomly chosen from (0, 1), and they have to meet another condition: *r*_1_ + *r*_2_ + *r*_3_ = 1; *x*_best_ is the global best solution of the entire population; the indices *a* and *b* are mutually exclusive integers randomly chosen from (1, 2,…, *N*), and they are different from the base index *i*. It is necessary to point out that *r*_1_, *r*_2_, and *r*_3_ are generated anew in each generation, but they are kept the same for all dimensions in each generation. Once the trial solution is generated, its associated food source has to compete with it for entering the next generation. It implies that the one with a better fitness value has the chance to survive.

Combining the above multiobjective strategies and the ABC algorithm, the basic flow of the EMOABC algorithm is shown in the following:

  Step 1: set the number of solution parameters (*D*), the number of populations (*N*), the maximum number of cycles (MNC), and “*limit*” value; randomly generate candidate solutions (**X** **=** [*x*_*ij*_]_*N*×*D*_).
  Step 2: calculate the fitness of each objective function, noninferior rank, and the crowding distance.
  Step 3: randomly select two solutions and choose the better storage solution. In this way, *N*/2 better solutions are selected.
  Step 4: search in the manner of equation (10) to produce *N*/2 solution, and if there is a solution beyond the boundary, it is placed on the boundary.
  Step 5: identify the better *N* solutions from the population of steps 3 and 4 according to noninferior rank and the crowding distance.
  Step 6: generate *N* new solutions by equation (15), and if there are any solutions beyond the boundary, they are placed on the tenth boundary.
  Step 7: select the better *N* solutions to form a new population according to noninferior rank and the crowding distance from the solutions in steps 1, 3, and 6.
  Step 8: determine if the termination condition is met; if so, output the Pareto front; otherwise, go to step 2.
  Step 9: arrange all solutions in the Pareto-optimal set, using equations (13) and (14), and then export a priority list of solutions.

### 3.3. Performance of the Proposed Algorithm

To verify the effectiveness of the EMOABC proposed in this paper, its performance is compared with those of NSGA-II and MOPSO. Convergence and diversity are usually chosen as evaluation criteria, and their specific mathematical expressions can be found in the literature [30, 31]. To ensure the fairness of algorithm testing, the size of the initial population *N* is set to 60 and the maximum number of cycles is 1000 for all algorithms on each test function. To achieve the best performance of the other two algorithms, their control parameters were set using the recommended values from the corresponding original literature. For EMOABC, the *limit* was set to 0.6 × *D* × *N*. To avoid the adverse effect of randomness on algorithm evaluation, each algorithm was run 30 times independently, and the mean value and the standard deviation of convergence and diversity were calculated, and the results of each algorithm for three benchmark functions ZDT1, ZDT2, and ZDT3 are shown in Table 1. Detailed expressions of ZDT1, ZDT2, and ZDT3 can be found in the literature [30]. Three algorithms have been run in MATLAB R2020a on a personal computer with Core 2 Duo 2.13 GHz processor and 4 GB memory.

From Table 1, the best values have been marked in bold. In terms of diversity, compared to other algorithms, the EMOABC algorithm obtained the most uniform Pareto front for each test problem with good distribution characteristics, indicating that the EMOABC algorithm has obvious advantages in distribution characteristics; in terms of convergence, for the ZDT3 problem, the EMOABC algorithm performs slightly worse than the NSGA-II algorithm but better than the MOPSO algorithm. Besides, the standard deviations of convergence and diversity obtained by the EMOABC algorithm are small, indicating that this algorithm is more stable and can almost always converge to the optimal nondominated frontier within the maximum number of cycles, which proves the effectiveness of the EMOABC algorithm to obtain a wider, uniform, and realistic Pareto solution set frontier.

Table 1 cannot completely reflect the results obtained by three algorithms; for this reason, and Figure 2 shows the noninferior optimal solution sets of three benchmark functions obtained by three algorithms.

As can be seen in Figure 2, the Pareto-optimal solutions of the EMOABC algorithm on ZDT1–3 can approximate the theoretical Pareto-optimal solution of each function very well, which has especially a good distribution. This experimental result once again verifies the effectiveness and advancement of the EMOABC algorithm for the multiobjective optimization problem.

## 4. Simulation and Discussion

The proposed method has been applied to two cases of mineral processing plants with different water sources and it is compared with MOPSO and NSGA-II to solve this problem. Parameters settings for three algorithms applied to two cases are the same as those set in Section 3.3.

### 4.1. Case 1

Case 1 is that the proposed algorithm is applied to the MPWD model based on mineral processing supplied by four water sources. The parameters about upper and lower limits for Case 1 are shown in Table 2, where 1 represents freshwater, 2 represents tailings water, 3 represents clean water, and 4 represents in-plant water. For recycled water, the lower cost with water source should be used first. In Case 1, since *c*_2_ < *c*_4_ < *c*_3_, set the penalty factor *α* = 3, *β* = 14, and *χ* = 8. The macro model, which uses historical data as a sample, is built by a stepwise regression approach [34]. The macro model of the water supply network and the macro model of the pressure control point in Case 1 are given in Tables 3 and 4, respectively. The following macro models (in Tables 3–6) are all simulation models.

To optimize both mineral processing water costs and the amount of recycled water simultaneously, the proposed EMOABC algorithm has been applied in the MPWD model with *q*_sum_ = 3000 and 4000. The five best solutions and best *ƞk* are summarized in Tables 7 and 8. The higher the value of *ƞk* for a solution, the higher the priority of the solution. From Table 7, we can see that *C* (**Q**) in *S*_2_ and *S*_3_ is slightly different, but *q*_1_–*q*_4_ in *S*_2_ and *S*_3_ are completely different. Also, the difference between *q*_1_–*q*_4_ in *S*_2_ and *S*_5_ is not significant, but the difference of *C* (*Q*) in *S*_2_ and *S*_5_ is obvious. The above denotes that a set of optimal solutions are obtained by the proposed EMOABC algorithm. The comparison between Tables 7 and 8 shows that when *q*_sum_ rises from 3000 to 4000, *q*_1_, *q*_2_, *q*_3_, and *q*_4_ increase accordingly, while *q*_3_ generally declines. *q*_2_ increases the most due to its low cost, and the decline in *q*_3_ is due to its high cost. The results of using EMOABC algorithm to schedule the flow of different water sources are consistent with those of manual regulation.

The MPWD model is solved using EMOABC, NSGA-II, and MOPSO. A comparison of the results obtained by three algorithms is shown in Table 9. It is seen that the EMOABC algorithm yields a lower cost of mineral processing water and a higher amount of recycled water (in bold) than the other two algorithms.

From Figure 3, it can be observed that EMOABC can discover a well-distributed and diverse solution set for this problem, while the other two algorithms only find some sparse distributions.

### 4.2. Case 2

Case 2 is that the proposed algorithm is applied to the MPWD model based on mineral processing supplied by six water sources. The parameters about upper and lower limits for Case 2 are shown in Table 10, where 1 represents freshwater no. 1, 2 represents freshwater no. 2, 3 represents tailings water no. 1, 4 represents tailings water no. 2, 5 represents clean water, and 6 represents in-plant water. For recycled water, the water source with a lower cost should be used first. In Case 2, since *c*_3_ < *c*_4_ < *c*_6_ < *c*_5_, set the penalty factor *α*_1_ = 3, *α*_2_ = 4, *β* = 14, and *χ* = 8. The macro model of the water supply network and the macro model of the pressure control point in Case 2 are given in Tables 5 and 6.

In this case, *C* (*Q*) and *M* (*Q*ʹ), two competing objectives, are optimized simultaneously by the EMOABC algorithm, and the five best solutions are shown in Tables 11 and 12. From Tables 11 and 12, the convergence of the solutions in Case 2 is as good as that in Case 1. It is worth noting that as the number of water sources increases, the water selection options are diverse. A comparison of the results obtained by MOPSO, NSGA-II, and EMOABC in Case 2 is shown in Table 13. From Table 13, we can observe that the EMOABC algorithm obtains the optimal solution (in bold) in Case 2 similar to Case 1.

Figure 4 shows the distribution of nondominated solutions obtained by NSGA-II, MOPSO, and EMOABC in Case 2. It is seen from them that EMOABC spreads well on the optimization problem, the function value obtained by EMOABC is significantly better than that obtained by NSGA-II, and MOPSO and EMOABC can find a better spread and more solutions in the entire Pareto-optimal region than the other two algorithms. It is indicated that the proposed algorithm is more effective than the other algorithms for solving the MPWD problem. Figures 3 and 4 also show that the two objectives of maximizing the amount of recycled water and minimizing mineral processing water costs conflict. As mineral processing water costs increase, the recycled water consumption decreases, and vice versa.

### 4.3. Algorithm Complexity Analysis

Complexity analysis of the above algorithms was performed using the time response for both cases. The average computation time for all algorithms over 30 runs is given in Table 14. From Table 14, it can be seen that EMOABC takes the most computation time. This can be explained by the fact that the multiple strategies integrated in EMOABC enhance the search capability at the cost of increased computation. In conclusion, EMOABC requires more computation time to achieve better results compared to other algorithms.

## 5. Conclusions

The main goal of this study was to solve the MPWD problem effectively. In this study, an MPWD optimization model was developed to maximize the amount of recycled water and minimize mineral processing water costs, with consideration of various constraints. To solve this multiobjective model, the EMOABC algorithm was proposed as an optimizer derived from the ABC algorithm. This study has shown that the developed model was theoretically valid and reasonable and could be utilized to provide decision support for actual MPWD. The study has also shown that the proposed algorithm is competent to solve the MPWD problem and is better than NSGA-II and MOPSO in both benchmark functions and cases.

A limitation of this study is that the developed model only has two objectives. The MPWD problem described as a three-objective or even four-objective model may be more realistic. Therefore, building a three-objective or even four-objective model for this MPWD problem is a matter of future work. Meanwhile, continued research of the multiobjective artificial bee colony (MOABC) algorithm is also a focus. In particular, aiming at a three-objective or even four-objective model for this MPWD problem, the concept of multihives bee will be introduced into the ABC algorithm to further improve the performance of the MOABC algorithm.

## Figures and Tables

**Figure 1:** The composition of water source in the mineral processing plant.

**Figure 2:** The comparable Pareto front obtained by three algorithms.

**Figure 3:** Pareto fronts obtained by NSGA-II, MOPSO, and EMOABC for *C* (*Q*) and *M* (*Q*ʹ) in Case 1.

**Figure 4:** Pareto fronts obtained by NSGA-II, MOPSO, and EMOABC for *C* (*Q*) and *M* (*Q*ʹ) in Case 2.

**Table 1:** The comparable results between EMOABC, NSGA-II, and MOPSO.

Criteria	Algorithm		ZDT1	ZDT2	ZDT3
Convergence	EMOABC	Mean	3.6239*e* − 3 2.3514*e* − 2	2.2485*e* − 2 2.6594*e* − 1	6.3256*e* − 2 2.6585*e* − 3
		Std			
	NSGA-II	Mean	3.9635*e* − 3 2.6985*e* − 2	2.9651*e* − 2 2.9985*e* − 1	5.5883*e* − 2 1.4154*e* − 3
		Std			
	MOPSO	Mean	4.1265*e* − 3 3.6517*e* − 2	2.8654*e* − 2 3.9914*e* − 1	7.9562*e* − 2 3.1953*e* − 3
		Std			
Diversity	EMOABC	Mean	6.6263*e* − 3	5.6156*e* − 2	3.6989*e* − 2
		Std	4.5696*e* − 4	4.2654*e* − 3	2.5359*e* − 3
	NSGA-II	Mean	3.3659*e* − 2	3.4889*e* − 1	3.7569*e* − 1
		Std	5.6387*e* − 2	3.1245*e* − 1	3.1245*e* − 2
	MOPSO	Mean	6.9159*e* − 2	7.6385*e* − 2	4.7646*e* − 1
		Std	5.4512*e* − 2	6.2589*e* − 3	3.6632*e* − 2

**Table 2:** Related parameters in Case 1.

Water sources	*q*_*i*_^min^ (m^3^/h)	*q*_*i*_^max^ (m^3^/h)	*p*_*i*_^min^ (MPa)	*p*_*i*_^max^ (MPa)	*h*_*i*_ (m)	*c*_*i*_ ($/m^3^)	cp_*i*_^min^ (MPa)
1	100	1000	0.15	0.95	15	0.11	0.13
2	120	3000	0.18	0.86	56	0.24	0.14
3	110	2000	0.17	0.93	26	0.46	0.13
4	95	1500	0.16	0.74	5	0.32	0.11

**Table 3:** Related macro model of water supply network in Case 1.

Water sources	*f*(*q*_sum_, *q*_*i*_, *q*_*i*_*q*_*j*_)	
1	0.145+2.618 × 10^−9^ × *q*_1_^2^+3.698 × 10^−9^ × *q*_3_^2^+6.594 × 10^−8^ × *q*_2_*q*_3_+2.365 × 10^−8^ × *q*_sum_^2^	
2	0.128+4.513 × 10^−9^ × *q*_1_^2^+6.485 × 10^−8^ × *q*_2_^2^+2.684 × 10^−10^ × *q*_1_*q*_2_+9.264 × 10^−10^ × *q*_sum_^2^	
3	0.117+1.561 × 10^−9^ × *q*_3_^2^+1.248 × 10^−9^ × *q*_4_^2^+5.654 × 10^−9^ × *q*_1_*q*_4_+4.589 × 10^−8^ × *q*_sum_^2^	
4	0.124+2.415 × 10^−9^ × *q*_4_^2^+8.261 × 10^−9^ × *q*_1_*q*_3_+1.368 × 10^−8^ × *q*_sum_^2^	

**Table 4:** Related macro model of the pressure control point in Case 1.

Water source	*f*′(*q*_sum_, *q*_*i*_)
1	0.109+1.529 × 10^−9^ × *q*_1_^2^+3.659 × 10^−10^ × *q*_sum_^2^
2	0.123+4.268 × 10^−8^ × *q*_2_^2^+5.364 × 10^−9^ × *q*_sum_^2^
3	0.151+7.268 × 10^−10^ × *q*_3_^2^+5.269 × 10^−8^ × *q*_sum_^2^
4	0.124+6.324 × 10^−8^ × *q*_4_^2^+8.624 × 10^−10^ × *q*_sum_^2^

**Table 5:** Related macro model of water supply network in Case 2.

Water sources	*f*(*q*_sum_, *q*_*i*_, *q*_*i*_*q*_*j*_)
1	0.125+3.584 × 10^−8^ × *q*_1_^2^+5.629 × 10^−10^ × *q*_2_^2^+2.598 × 10^−9^ × *q*_3_*q*_4_+4.268 × 10^−9^ × *q*_sum_^2^
2	0.114+8.268 × 10^−10^ × *q*_2_^2^+3.628 × 10^−9^ × *q*_6_^2^+6.324 × 10^−9^ × *q*_3_*q*_5_+8.529 × 10^−10^ × *q*_sum_^2^
3	0.115+1.269 × 10^−8^ × *q*_3_^2^+1.562 × 10^−8^ × *q*_6_^2^+4.263 × 10^−9^ × *q*_4_*q*_5_+9.264 × 10^−10^ × *q*_sum_^2^
4	0.142+7.261 × 10^−9^ × *q*_4_^2^+6.826 × 10^−9^ × *q*_1_^2^+5.987 × 10^−9^ × *q*_1_*q*_3_+8.154 × 10^−10^ × *q*_sum_^2^
5	0.138+9.261 × 10^−10^ × *q*_5_^2^+5.698 × 10^−10^ × *q*_2_^2^+4.358 × 10^−9^ × *q*_3_*q*_6_+7.569 × 10^−9^ × *q*_sum_^2^
6	0.152+3.652 × 10^−8^ × *q*_6_^2^+1.268 × 10^−8^ × *q*_2_*q*_4_+2.584 × 10^−9^ × *q*_sum_^2^

**Table 6:** Related macro model of the pressure control point in Case 2.

Water source	*f*′(*q*_sum_, *q*_*i*_)
1	0.121+2.316 × 10^−10^ × *q*_1_^2^+8.362 × 10^−9^ × *q*_sum_^2^
2	0.132+5.326 × 10^−9^ × *q*_2_^2^+3.958 × 10^−10^ × *q*_sum_^2^
3	0.142+9.635 × 10^−10^ × *q*_3_^2^+4.369 × 10^−9^ × *q*_sum_^2^
4	0.129+2.589 × 10^−8^ × *q*_4_^2^+5.241 × 10^−10^ × *q*_sum_^2^
5	0.161+7.125 × 10^−9^ × *q*_5_^2^+8.629 × 10^−10^ × *q*_sum_^2^
6	0.135+5.264 × 10^−9^ × *q*_6_^2^+1.259 × 10^−8^ × *q*_sum_^2^

**Table 7:** Five best solutions for Case 1 using the EMOABC (*q*_sum_ = 3000).

Solutions	*q*_1_ (m^3^/h)	*q*_2_ (m^3^/h)	*q*_3_ (m^3^/h)	*q*_4_ (m^3^/h)	*C* (*Q*) ($/h)	*M* (*Q*ʹ) (m^3^/h)	*ƞk*
*S*_1_	328	1156	875	641	61577	20084	0.0536
*S*_2_	396	1297	801	506	61683	19153	0.0534
*S*_3_	298	1307	783	612	61681	19779	0.0531
*S*_4_	384	1376	752	488	61613	18560	0.0529
*S*_5_	395	1298	803	504	61756	19168	0.0528

**Table 8:** Five best solutions for Case 1 using the EMOABC (*q*_sum_ = 4000).

Solutions	*q*_1_ (m^3^/h)	*q*_2_ (m^3^/h)	*q*_3_ (m^3^/h)	*q*_4_ (m^3^/h)	*C* (*Q*) ($/h)	*M* (*Q*ʹ) (m^3^/h)	*ƞk*
*S*_1_	422	2120	804	654	103820	22848	0.0546
*S*_2_	439	2206	739	616	103450	21892	0.0554
*S*_3_	432	2072	824	672	103380	23128	0.0562
*S*_4_	398	2218	730	654	103580	22106	0.0558
*S*_5_	406	2195	752	647	103790	22289	0.0549

**Table 9:** The best solutions for Case 1 using three algorithms.

	MOPSO		NSGA-II		EMOABC	
	*q*_sum_ = 3000	*q*_sum_ = 4000	*q*_sum_ = 3000	*q*_sum_ = 4000	*q*_sum_ = 3000	*q*_sum_ = 4000
*q*_1_	395	419	329	395	384	432
*q*_2_	1294	2118	1159	2221	1376	2082
*q*_3_	802	807	864	732	752	794
*q*_4_	509	656	648	652	488	692
*C* (*Q*)	61668	103900	61641	103750	**61577**	**103380**
M (Qʹ)	19182	22900	20057	22127	**20084**	**23128**

Bold highlights that the algorithm proposed in this paper achieves better results.

**Table 10:** Related parameters in Case 2.

Water sources	*q*_*i*_^min^ (m^3^/h)	*q*_*i*_^max^ (m^3^/h)	*p*_*i*_^min^ (MPa)	*p*_*i*_^max^ (MPa)	*h*_*i*_ (m)	*c*_*i*_ ($/m^3^)	cp_*i*_^min^ (MPa)
1	110	900	0.16	0.96	12	0.12	0.14
2	100	800	0.19	0.87	23	0.13	0.15
3	120	2500	0.18	0.92	45	0.24	0.16
4	105	2800	0.17	0.76	56	0.26	0.13
5	130	1200	0.15	0.85	25	0.48	0.17
6	115	950	0.14	0.63	3	0.33	0.14

**Table 11:** Five best solutions for Case 2 using EMOABC (*q*_sum_ = 5000).

Solutions	*q*_1_ (m^3^/h)	*q*_2_ (m^3^/h)	*q*_3_ (m^3^/h)	*q*_4_ (m^3^/h)	*q*_5_ (m^3^/h)	*q*_6_ (m^3^/h)	*C* (*Q*) ($/h)	*M* (*Q*ʹ) (m^3^/h)	*ƞk*
*S*_1_	218	324	1487	1295	894	692	80912	27693	0.0585
*S*_2_	352	415	1352	1415	841	625	80005	26490	0.0587
*S*_3_	364	325	1238	1449	828	814	80087	27614	0.0596
*S*_4_	316	348	1336	1479	779	742	80049	26766	0.0594
*S*_5_	355	362	1302	1209	893	879	79153	28276	0.0598

**Table 12:** Five best solutions for Case 2 using EMOABC (*q*_sum_ = 6000).

Solutions	*q*_1_ (m^3^/h)	*q*_2_ (m^3^/h)	*q*_3_ (m^3^/h)	*q*_4_ (m^3^/h)	*q*_5_ (m^3^/h)	*q*_6_ (m^3^/h)	*C* (*Q*) ($/h)	*M* (*Q*ʹ) (m^3^/h)	*ƞk*
*S*_1_	402	406	1789	1703	906	794	102800	31215	0.0642
*S*_2_	421	456	1859	1906	806	552	102540	28901	0.0649
*S*_3_	359	396	1952	1589	863	841	102300	31022	0.0651
*S*_4_	398	412	1652	1856	786	896	102240	31272	0.0648
*S*_5_	416	395	1742	1647	911	889	102230	31680	0.0654

**Table 13:** The best solutions for Case 2 using three algorithms.

	MOPSO		NSGA-II		EMOABC	
	*q*_sum_ = 5000	*q*_sum_ = 6000	*q*_sum_ = 5000	*q*_sum_ = 6000	*q*_sum_ = 5000	*q*_sum_ = 6000
*q*_1_	322	415	388	429	355	416
*q*_2_	405	323	361	398	362	395
*q*_3_	1212	1842	1251	1662	1302	1742
*q*_4_	1315	1772	1289	1731	1209	1647
*q*_5_	881	845	896	919	893	911
*q*_6_	865	803	815	861	879	889
*C* (*Q*)	79379	102960	79398	102550	**79153**	**102230**
*M* (*Q*ʹ)	28150	30868	27973	31664	**28276**	**31680**

Bold highlights that the algorithm proposed in this paper achieves better results.

**Table 14:** Computing time of all algorithms for both cases.

	Computing time (s)		
	EMOABC	NSGA-II	MOPSO
Case 1	58.6	40.2	47.8
Case 2	74.4	59.5	64.7

## Data Availability

No data were used to support this study.
